The article "Effects of Treadmill Exercise on Mitochondrial DNA Damage and Cardiomyocyte Telomerase Activity in Aging Model Rats Based on Classical Apoptosis Signaling Pathway" was retracted in 2023. Reasons: unreliable results or conclusions; concerns about the data; concerns about the peer review; concerns about the citations.

# Effects of Treadmill Exercise on Mitochondrial DNA Damage and Cardiomyocyte Telomerase Activity in Aging Model Rats Based on Classical Apoptosis Signaling Pathway

**DOI:** 10.1155/2022/3529499

**Published:** 2022-04-14

**Authors:** Chao Liang, Xiaoli Zhou, Meiling Li, Zhengpeng Song, Jinyan Lan

**Affiliations:** ^1^School of Martial Arts, Wuhan Sports University, Wuhan 430079, China; ^2^Shanxi Traditional Chinese Medical Hospital, Taiyuan 030012, China; ^3^College of Physical Education, Shanxi University, Taiyuan 237016, China

## Abstract

In order to explore the effect of treadmill exercise on mitochondrial DNA damage and myocardial telomerase activity in aging model rats based on the classical apoptosis signaling pathway, a total of 36 clean-grade male SD rats are selected. After modeling, the rats are randomly divided into groups, namely, control and 3 times/w and 6 times/w exercise rats, with 12 rats in each group. After the rats of each group are modeled, the myocardial tissue and cells are collected, the apoptosis of myocardial cells is detected by TUNEL method, and the protein expressions of Bax and Bcl-2 in myocardial tissue are detected by western blotting. The mtDNA content of the control rats is the highest, which is significantly higher than that of the exercise group (*P* < 0.05); the expression of mtDNA content in the heart of the rats exercising 3 times/w is significantly higher than that of the rats exercising 6 times/w (*P* < 0.05); cardiomyocyte apoptosis AI value, Bcl-2, and Bax expressions of the control rats is the highest and significantly higher than those in the exercise group (*P* < 0.05); Bcl-2/Bax in the control rats is the lowest and is significantly lower than that in the exercise group (*P* < 0.05). The AI value, Bcl-2, and Bax expression of myocardial cell apoptosis in 3 times/w exercise rats are significantly higher than those in 6 times/w exercise rats (*P* < 0.05); Bcl-2/Bax of 3 times/w exercise rats is significantly lower than that in 6 times/w exercise rats (*P* < 0.05); by observing the rats that completed treadmill exercise, Akt2 protein of 3 times/w exercise rats and 6 times/w exercise rats is observed and analyzed. Compared with the control rats, the expressions of the two proteins are increased in 3 times/w exercise rats and 6 times/w exercise rats, and the upregulation in 6 times/w exercise rats is significantly increased and higher than that in 3 times/w exercise rats (*P* < 0.05). For aging rats, treadmill exercise can reduce the body Bcl-2 and Bax values, improve the mitochondrial DNA damage and myocardial cell telomerase activity in aging model rats, and slow down the aging process.

## 1. Introduction

Aging is a process in which the physiological functions of the body gradually decline with age and eventually die. Some studies have shown that the occurrence of apoptosis has a negative impact on aging mainly by destroying important non-regenerative cells [1, 2]. With the occurrence of aging, the apoptosis of various tissues and organs such as cardiac muscle, brain tissue, and adrenal gland will increase excessively, thereby promoting the aging process to a certain extent [3]. Therefore, reducing or inhibiting excessive apoptosis in aging organisms and increasing corresponding interventions may help to delay aging [4–6]. In addition, from the perspective of the mechanism of apoptosis, the process is mainly controlled by genes. An active death of cells plays an important role in the occurrence, development, proliferation, and differentiation of intracellular apoptosis and plays an important role in the changes of diseases and the process of aging [7]. With the occurrence of aging, it will further lead to the decline of the corresponding functions of tissues and organs, thereby aging the aging process. The direct line of mitochondrial DNA (mitochondria DNA, mtDNA) belongs to maternal inheritance [8]. No matter in which cell, there is a close relationship between DNA copy data and tissue [9]. A number of research studies have shown that cardiac aging is often accompanied by a general decline in mitochondrial function, expansion of dysfunctional mitochondrial clones, increased reactive oxygen species (ROS) production, inhibition of mitochondrial autophagy, and dysregulation of mitochondrial quality control processes [10]. Therefore, a comprehensive understanding of the regulatory role of mitochondria in cardiac aging and the search for new therapeutic approaches to mitigate mitochondrial damage and restore collective mitochondrial viability are expected to reduce the morbidity and mortality associated with cardiac aging and slow down the aging process. A multitude of empirical studies have demonstrated that long-term regular aerobic exercise not only lowers blood pressure but also has the ability to improve the structure and function of the heart, such as improving pathological myocardial hypertrophy and myocardial fibrosis leading to ventricular remodeling. FENG et al.'s study demonstrated that 4 weeks of table running exercise had a significant protective effect on myocardial injury in rats [11]. However, the specific molecular mechanisms of the effects of exercise on myocardial remodeling and cardiac function need further in-depth study. Based on this, this experiment took the aging model rats as the experimental objects and grouped the experimental rats according to the frequency of treadmill exercise in different degrees and explored the effect of treadmill exercise on mitochondrial DNA damage, myocardial damage, and effects of cellular telomerase activity in the aging model rats based on the classical apoptosis signaling pathway.

The article "Effects of Treadmill Exercise on Mitochondrial DNA Damage and Cardiomyocyte Telomerase Activity in Aging Model Rats Based on Classical Apoptosis Signaling Pathway" was retracted in 2023. Reasons: unreliable results or conclusions; concerns about the data; concerns about the peer review; concerns about the citations.

The rest of the paper is structured as follows.  Section 2 provides method of this research. Methodology covering both data collection is described in Section 3. Detection of Bax, Bcl-2, and other protein expressions in myocardial tissue by immunoblotting is described in Section 4. The data analysis is described in Section 5.  Section 6 presents the results of this research. This is followed by discussion which includes implications and limitations and conclusion in Section 7.

## 2. The Experimental Method

A total of 36 clean-grade male SD rats are selected, with a body weight of 195-263 g, an average of 256.93 ± 21.52 g, and an 8-week-old animal. The animals are provided by Tianqin Biological Company.

Apoptosis detection kit is purchased from ITC, USA; Bcl-2 I antibody is purchased from Netics, USA; horseradish peroxidase- (HRP-) labeled goat anti-rabbit secondary antibody is purchased from CST Company in the United States; the luminescent agent, model ECL-plus, is purchased from Amersham Biosciences; the protein lysate is purchased from Shanghai Biyuntian Institute of Biotechnology.

According to the national rodent standard, the rats are fed with natural circadian lighting and allowed to eat freely [12–14]. All rats are placed in a room temperature environment of 24°C, the operation light time is 12 hand, and the humidity is set to about 50%. First, all rats are fed for one week, and the feeding method is adaptive feeding. D-galactose and normal saline are mixed to prepare a 5% concentration injection. The model rats are injected with subcutaneous injection at a dose of 500 mg/kg/d for 6 weeks. After the modeling is completed, the rats are randomly divided into groups, namely, control and 3 times/w and 6 times/w exercise rats, 12 rats in each group. The treadmill exercise intervention program was based on existing studies [15–18]. The training time was selected in the dark period (18:00~20:00) and adjusted according to the specific conditions of animal movement. In the first week, rats exercised at a speed of 8.0-15 m/min for 15-20 min. In the second week, rats exercised at a speed of 15 m/min for 30-45 min. From the 3rd to the 12th week, the above exercise speed and frequency remained unchanged. All exercise rats underwent 12 w training. Eight rats are randomly selected and sacrificed from the three groups [19, 20]. All rats are fasted for 12 hours before sacrifice. The myocardial tissue of the left ventricular free wall of the rats is collected, and the apoptosis of cardiomyocytes is performed by a TUNEL method [21].

The article "Effects of Treadmill Exercise on Mitochondrial DNA Damage and Cardiomyocyte Telomerase Activity in Aging Model Rats Based on Classical Apoptosis Signaling Pathway" was retracted in 2023. Reasons: unreliable results or conclusions; concerns about the data; concerns about the peer review; concerns about the citations.

After the rats of each group completed the modeling, the rats should be anesthetized immediately. The anesthetic drug is sodium pentobarbital with a concentration of 2%. Rats are killed. Use sterile scissors to cut the edges of the left and right ribs of the rat until they reach the abdominal wall of the rat, turn the ribs to the head side along the front sides of the abdominal wall of the rat, and place the heart root of the rat. Keep the artery, wait for the heart to be cut at 3-4 mm, and take out the heart quickly; after taking out the rat's heart, it is quickly dissected from top to bottom, and the myocardial tissue near the apex is separated; about 2 mg is enough. The myocardial tissue used in this experiment is this part. It should be noted that the above operation steps should be completed within 10 minutes. After completion, the fat and connective tissue in the heart should be carefully removed and then placed in PBS lysis solution at 0°C. The remaining myocardial tissue should be carefully stored in a liquid nitrogen tank and placed in a low-temperature refrigerator. After the material is collected, the steps in the refrigerator should be completed within 5 minutes.

## 3. TUNEL Assay to Detect Cardiomyocyte Apoptosis

First, the hydrogen peroxide is prepared, and the concentration is set to 3%. The myocardial tissue slices are taken and treated with hydrogen peroxide for 10 minutes. Then, the labeled buffer is added to the slices, and they are placed in an environment at room temperature of 37°C for 2 hours. The blocking solution completes the blocking, and then it is placed at room temperature. After 30 minutes, biotinylated antibodies are added to the slices to allow them to react with each other for 30 minutes and placed in an environment where the room temperature is 37°C; finally, the reaction of the dilution solution is completed. For color development, ABC is used as the diluent, and a series of operations such as hematoxylin counterstaining, dehydration, and mounting are performed and finally placed under a microscope for observation. Observing the cell state and color under the microscope: if the cardiomyocytes are blue, it is normal; if the cardiomyocytes are brown, it is positive for apoptosis. The rats are examined and processed for two slices, and each slice is placed under a ×400 field of view to detect the number of apoptotic cells: apoptosis index = positive number of apoptotic cells/total number of cells × 100% [22].

## 4. Detection of Bax, Bcl-2, and Other Protein Expressions in Myocardial Tissue

First, the myocardial samples of each group are extracted with a mass of 100 mg, and then RIPA lysate is added to the cells of each group to extract the total protein of the cells. The protein concentration is detected using the BCA kit. After the detection, the samples are subjected to SDS-PAGE, the protein gel is separated, and it is placed in a PVDF membrane for blocking treatment. The selected antibodies included Bax monoclonal antibody, and mouse anti-Bcl-2 needs to be placed at room temperature for 1 h, washed with TBST, and then developed, using ECL as a developer and using ImageJ software to analyze its gray value [23]. At the same time, the internal reference is set to *β*-actin; the target protein band and the *β*-actin band are obtained by the same electrophoresis, and the ratio of the two is used as a quantitative reference.

The article "Effects of Treadmill Exercise on Mitochondrial DNA Damage and Cardiomyocyte Telomerase Activity in Aging Model Rats Based on Classical Apoptosis Signaling Pathway" was retracted in 2023. Reasons: unreliable results or conclusions; concerns about the data; concerns about the peer review; concerns about the citations.

## 5. The Data Analysis

In this study, all the data are organized, and a corresponding database is established for it, and all the databases are entered into SPSS 26.0 for neutral data processing, in which the measurement data is tested for normality, expressed as *x* ± *s*, a multigroup test is *F* for normality for between groups, and the Mann–Whitney *U* test for non-normality; the rate is expressed as%, and the test is *χ*^2^. When *P* < 0.05, the difference between the data is statistically significant.

## 6. The Experimental Result

### 6.1. Comparison of Mitochondrial DNA Content of Rats in Each Group

The mtDNA content of the control rats is the highest, which is significantly higher than that of the exercise group (*P* < 0.05); the expression of mtDNA content in the hearts of the rats exercising 3 times/w is significantly higher than that of the rats exercising 6 times/w (*P* < 0.05), as shown in Table 1.

### 6.2. Cardiomyocyte Apoptosis and Detection Results of Bcl-2 and Bax

The apoptosis value of cardiomyocytes and the expression of Bcl-2 and Bax in the control rats are the highest and are significantly higher than those in the exercise group (*P* < 0.05); the Bcl-2/Bax in the control rats is the lowest and is significantly lower than that in the exercise rats (*P* < 0.05); the apoptosis value of cardiomyocytes and the expression of Bcl-2 and Bax in 3 times/w exercise rats are significantly higher than those in 6 times/w exercise rats (*P* < 0.05); Rat Bcl-2/Bax of 3 times/w exercise rats is significantly lower than that of 6 times/w exercise rats (*P* < 0.05).  Table 2 shows the comparison of cardiomyocyte apoptosis results.  Table 3 shows the expression analysis of Bcl-2 and Bax results in cardiomyocytes.  Figure 1 presents TUNEL staining results of three groups of rat cardiomyocytes.  Figure 2 displays the results of Bcl-2 and Bax immunoblotting in three groups of rat cardiomyocytes.

The article "Effects of Treadmill Exercise on Mitochondrial DNA Damage and Cardiomyocyte Telomerase Activity in Aging Model Rats Based on Classical Apoptosis Signaling Pathway" was retracted in 2023. Reasons: unreliable results or conclusions; concerns about the data; concerns about the peer review; concerns about the citations.

### 6.3. Results of Myocardial Total RNA and Internal Reference Gene in Three Groups of Rats

The rat myocardial total RNA integrity and electrophoresis detection are good, and the RT-PCR internal reference gene amplification curve and dissolution curve are completed.  Figure 3 shows the total RNA integrity and electrophoresis detection.  Figure 4 is the amplification curve of RT-PCR internal reference gene.

### 6.4. Comparison of Myocardial PPAR Q and Akt2 Expression Results

By observing the rats that completed the treadmill exercise, it is found that compared with the control rats, the expressions of *ΔΔ*cT and 2-AACT are upregulated in the 3 times/w exercise rats and the 6 times/w exercise rats, and the upregulation amplitude of 6 times/w exercise rats is significantly higher than that of 3 times/w exercise rats (both *P* < 0.05). The expressions of the two proteins are increased in both 3times/w exercise rats and 6 times/w exercise rats, and the upregulation range of 6 times/w exercise rats is significantly higher than that of 3 times/w exercise rats (both *P* < 0.05).  Table 4 shows the expression analysis of PPAR Q and Akt2 results in cardiomyocytes.  Figure 5 is the expression results of myocardial PPAR Q and Akt2 in the three groups.  Figure 6 is expression map of myocardial PPAR Q and Akt2 protein in three groups.

## 7. Discussion and Conclusion

### 7.1. Discussion

From the perspective of modern science, aging is a very normal phenomenon in the process of human evolution [24–26]. In other words, aging is a passive by-product of the body in the process of human evolution. Senescent cells continue to differentiate, thus changing their state, resulting in a gradual slowdown in their proliferation ability, and even partial loss of proliferation ability, resulting in overall body function and tissue decline [27]. From the performance of aging, the changes in the form and function of the motor system are one of the changes that can be closely observed. The change of system morphology and function is a relatively complex process, so it is extremely important to study the relationship between exercise and aging [28, 29].

Essentially, mitochondria, as the DNA of an organism, is a double-stranded circular molecule that contains hundreds of copies in cells [30]. Since the early 1980s, the relationship and theoretical knowledge between mtDNA free radicals and aging have been affirmed by most scholars [31, 32]. The theory points out that if oxidative damage occurs in the body, under the intervention of mtDNA, mitochondrial function may be hindered, which in turn leads to a vicious circle, which seriously threatens and affects the occurrence and development of aging [33, 34]. Mitochondria are the regulation center of apoptosis, and Cyt C, a key molecule, is a protein encoded by cytosolic genes whose release mediates the apoptotic pathway relevant to the regulatory control of Bcl-2 family members. Stimulation by apoptosis (damage to DNA, growth factor deficiency, etc.) causes Bax/Bak to form an oligomeric complex that inserts into the extramitochondrial membrane pore, leading to changes in mitochondrial osmotic pressure and loss of transmembrane potential, prompting the release of Cyt C from mitochondria to the cytoplasm, and binding to apoptosis activator 1 (Apaf-1) to form an apoptotic complex that activates Caspase-9 precursor, which in turn activates Caspase-3 and Caspase-7, triggers the Caspase cascade reaction, and thus induces apoptosis. During this period, other proapoptotic proteins such as Smac, Omi, and ARTS inhibit IAPs and contribute together to the apoptotic response [35]. In this experiment, it is found that the mtDNA content of the control rats is the highest, which is significantly higher than that of the exercise group (*P* < 0.05). The AI value of apoptosis in rat cardiomyocytes is the highest and is significantly higher than that in the exercise group (*P* < 0.05). When the body undergoes oxidative stress, mtDNA will be greatly damaged. If mtDNA damage is not repaired and alleviated in time, it may cause its mutation, and under the intervention of the electron transport chain, it may promote phosphorylation damage, reduce the functional efficiency of ETC, and cause the body to gradually reduce ATP production. Consistent with the research of Yoo et al., the scholars believe that in the process of body aging, mitochondrial DNA may mutate, thereby directly or indirectly affecting the occurrence of aging [35]. The main reason for the analysis is that the main location of mitochondrial DNA in the body is under the inner mitochondrial membrane of high oxygen free radicals, but because it cannot repair and deal with damaged tissues, mtDNA is prone to oxidative damage and even causes mutations. At present, the changes of mitochondrial DNA are mainly due to the increase and accumulation of DNA mutations and oxidative modifications with age [36]. In later tissues, the mitotic process is more pronounced after DNA changes, thus affecting body functions, reduce the body function, causing the occurrence of aging.

The article "Effects of Treadmill Exercise on Mitochondrial DNA Damage and Cardiomyocyte Telomerase Activity in Aging Model Rats Based on Classical Apoptosis Signaling Pathway" was retracted in 2023. Reasons: unreliable results or conclusions; concerns about the data; concerns about the peer review; concerns about the citations.

There is also a significant relationship between exercise and apoptosis of cardiomyocytes. This process is mainly affected by gene regulation. In the process of apoptosis, the Bcl-2 protein family plays an important role [37, 38]. The 2 family is divided into two categories; that is, one is antiapoptotic, mainly including Bal-2, Bcl-W, and CED9. The other is the promotion of cell death, including Bax, Bel-XS, and Bid. The Bcl-2 family proteins act on mitochondria by two main mechanisms: first, members of the Bcl-2 family proteins are able to precisely regulate the open state of MPTP; second, they induce the generation of new mitochondrial permeability pore channels. Both pathways result in the release of cytochrome C and apoptosis-inducing factors, etc. from the cytosolic intermembrane lumen into the cytosol. Cytochrome C activates apoptotic protease activating factor-1 (Apaf-1) and forms apoptotic vesicles with Apaf-1 and ATP, which accumulate in the cytosol. It activates Caspase-9 and binds to it to form an apoptotic complex, which in turn activates Caspase-3, which hydrolyzes various cellular constituents and causes apoptosis; it can directly reach the nucleus and cause chromosome aggregation and nuclear fragmentation, thus causing mitochondria-mediated apoptosis. In this experiment, it is found that the expression of apoptosis Bcl-2 and Bax in cardiomyocytes of the control rats is the highest and significantly higher than that of the exercise group (*P* < 0.05); the expression of apoptosis Bcl-2 and Bax in cardiomyocytes of 3 times/w exercise rats is significantly higher than that of 6 times/w exercise rats (*P* < 0.05); Bcl-2/Bax of 3 times/w exercise rats is significantly lower than that of 6 times/w exercise rats (*P* < 0.05); on the whole, in the process of apoptosis, Bcl-2 and Bax play an important role in a pair of functional genes, and their expression levels are related to apoptosis [39]. There is a significant correlation between the regulations of the pathway. When the expression of Bax is increased, the apoptosis of the body will be greatly deepened, and when the expression of Bcl-2 is increased, the apoptosis will be inhibited to a certain extent. However, studies usually use the ratio of Bcl-2 and Bax as the main reason for evaluating the strength of apoptosis inhibition [40, 41]. Compared with control rats, the protein expressions of *ΔΔ*cT, 2-AACT, PPAR Q, and Akt2 are all upregulated in 3 times/w exercise rats and 6 times/w exercise rats, and the upregulation range in 6 times/w exercise rats is significantly higher than that in 3 times/w exercise rats (all *P* < 0.05). Cardiomyocytes belong to an undifferentiated cell, although this cell is a mature cell, but it does not have the ability to proliferate [42, 43]. The apoptosis of cardiomyocytes may reduce the number of cells, and its cardiac function and myocardial tissue capacity will be significantly reduced, gradually turning to pathological development; that is, if cardiomyocytes undergo excessive apoptosis, the aging process of the heart may be accelerated [44, 47, 48]. Although this experiment has achieved certain results, there are still some deficiencies. There is a broad consensus on the central role of mitochondrial dysfunction. Because cardiomyocytes may be affected by various factors and mechanisms linking flawed mitochondrial quality control mechanisms (protein stabilization, biogenesis, kinetics, and autophagy) to dysfunctional organelles in the context of cardiac aging.

The article "Effects of Treadmill Exercise on Mitochondrial DNA Damage and Cardiomyocyte Telomerase Activity in Aging Model Rats Based on Classical Apoptosis Signaling Pathway" was retracted in 2023. Reasons: unreliable results or conclusions; concerns about the data; concerns about the peer review; concerns about the citations.

### 7.2. Conclusion

This study explores the effect of treadmill exercise on mitochondrial DNA damage and myocardial telomerase activity in aging model rats based on the classical apoptosis signaling pathway; a total of 36 clean-grade male SD rats are selected. After modeling, the rats are randomly divided into groups, namely, control and 3 times/w and/6 times/w exercise rats, with 12 rats in each group and carry out 12-week treadmill exercise intervention. At the current experimental settings, for aging rats, treadmill exercise can reduce the Bcl-2 and Bax values, improve mitochondrial DNA damage and myocardial cell telomerase activity in aging model rats, and alleviate the aging process.

## Figures and Tables

**Figure 1:** TUNEL staining results of three groups of rat cardiomyocytes (×400): (a) the control group; (b) the 3 times/w exercise group; (c) 6 times/w exercise group.

**Figure 2:** The results of Bcl-2 and Bax immunoblotting in three groups of rat cardiomyocytes: (a) the control group; (b) the 3 times/w exercise group; (c) the 6 times/w exercise group.

**Figure 3:** Total RNA integrity and electrophoresis detection.

**Figure 4:** Amplification curve of RT-PCR internal reference gene.

**Figure 5:** The expression results of myocardial PPAR Q and Akt2 in the three groups.

**Figure 6:** Expression map of myocardial PPAR Q and Akt2 protein in three groups.

**Table 1:** Comparison of mitochondrial DNA content of rats in each group.

Group	*n*	mtDNA (*μ*g/mL)
Control	12	4.32 ± 0.71
3 times/w exercise	12	2.32 ± 0.47
6 times/w exercise	12	1.51 ± 0.31
*F*		8.263
*P*		<0.001

Note: ∗ means compared with the control group; & means compared with 3 times/w exercise < 0.05.

**Table 2:** Comparison of cardiomyocyte apoptosis results.

Group	Apoptosis (%)
Control	36.03 ± 1.46
3 times/w exercise	27.89 ± 1.35^∗^
6 times/w exercise	24.35 ± 1.33^∗,&^
*F*	7.656
*P*	<0.001

**Table 3:** Expression analysis of Bcl-2 and Bax results in cardiomyocytes.

Group	Bcl-2	Bax	Bcl-2/Bax
Control	7.86 ± 0.92	2.23 ± 0.29	3.62 ± 0.18
3 times/w exercise	10.03 ± 0.56^∗^	1.92 ± 0.29^∗^	5.34 ± 0.36^∗^
6 times/w exercise	10.53 ± 0.75^∗,&^	1.81 ± 0.22^∗,&^	5.79 ± 0.51^∗,&^
*F*	6.529	11.256	8.771
*P*	<0.001	<0.001	<0.001

Note: ∗ means compared with the control group; & means compared with 3 times/w exercise < 0.05.

The article "Effects of Treadmill Exercise on Mitochondrial DNA Damage and Cardiomyocyte Telomerase Activity in Aging Model Rats Based on Classical Apoptosis Signaling Pathway" was retracted in 2023. Reasons: unreliable results or conclusions; concerns about the data; concerns about the peer review; concerns about the citations.

**Table 4:** Expression analysis of PPAR Q and Akt2 results in cardiomyocytes.

Group	PPAR Q	Akt2
Control	19.25 ± 0.85	11.16 ± 0.87
3 times/w exercise	32.26 ± 0.99^∗^	26.63 ± 1.59^∗^
6 times/w exercise	36.58 ± 1.24^∗,&^	54.85 ± 2.38^∗,&^
*F*	12.569	15.423
*P*	<0.001	<0.001

Note: ∗ means compared with the control group; & means compared with 3 times/w exercise < 0.05.

## Data Availability

The simulation experiment data used to support the findings of this study are available from the corresponding author upon request.
